The article "CT Signs and Differential Diagnosis of Peripheral Lung Cancer and Inflammatory Pseudotumor: A Meta-Analysis" was retracted in 2023. Reasons: signs of a paper mill; suspected computer-generated content; unreliable results or conclusions; concerns about the data.

# CT Signs and Differential Diagnosis of Peripheral Lung Cancer and Inflammatory Pseudotumor: A Meta-Analysis

**DOI:** 10.1155/2022/3547070

**Published:** 2022-01-03

**Authors:** Shiyi Zheng, Jie Shu, Jianan Xue, Caiyun Ying

**Affiliations:** ^1^Department of Radiology, The First People's Hospital of Chongqing Liang Jiang New Area, Chongqing, China; ^2^Department of Surgery, Xiangya Hospital, Central South University, Changsha, Hunan, China; ^3^Department of Ultrasound, China-Japan Union Hospital of Jilin University, Changchun, Jilin, China

## Abstract

We aimed to systematically evaluate the imaging features of peripheral lung cancer and inflammatory pseudotumor. PubMed, Embase, Cochrane Library, Chinese Knowledge Infrastructure (CNKI), Wanfang database (Wanfang), and Chinese Biomedical Network (CBM) were searched to collect relevant studies on CT image comparison of peripheral lung cancer and inflammatory pseudotumor. The search time was from database establishment to July 15, 2021. The search language was limited to Chinese and English. Data from the literature were screened and extracted, and meta-analysis was performed using Stata 16.0 software. A total of 8 cohort studies were included in this meta-analysis, including 675 patients. Meta-analysis showed that the lesion size of inflammatory pseudotumor was greater than that of peripheral lung cancer, and the difference had statistical significance [SMD = 0.29, 95% CI (0.01, 0.58), *P* < 0.05]. The difference in HU value between inflammatory pseudotumor and peripheral lung cancer CT had no statistical significance [SMD = −0.09, 95% CI (−0.79, 0.60), *P* > 0.05]. The HU value of enhanced CT of inflammatory pseudotumor was higher than that of peripheral lung cancer, and the difference had statistical significance [SMD = 0.75, 95% CI (0.15, 1.34), *P* < 0.05]. The incidence of calcification of inflammatory pseudotumor was significantly higher than that of peripheral lung cancer, and the difference had statistical significance [RR = 2.85, 95% CI (1.33, 6.11), *P* < 0.05]. The incidence of long hair puncture sign of inflammatory pseudotumor was lower than that of peripheral lung cancer, and the difference had statistical significance [RR = 0.49, 95% CI (0.24, 0.97), *P* < 0.05]. There was no significant difference between inflammatory pseudotumor and peripheral lung cancer in terms of cavity incidence, vacuole sign, pleural indentation, and bronchial inflation sign (*P* > 0.05). Based on the available literature evidence, it can be found that there are differences in the CT signs between peripheral lung cancer and inflammatory pseudotumor, and the lesion size, HU value on enhanced CT, incidence of calcification, and incidence of burr sign may be important indicators for differentiating peripheral lung cancer from inflammatory pseudotumor.

## 1. Introduction

Lung cancer is one of the most common malignant tumors and has become one of the leading causes of cancer death worldwide, mainly divided into central, peripheral, and diffuse lung cancer [1, 2]. Among them, peripheral lung cancer refers to lung cancer that occurs in the bronchi below the lung segment and is mainly seen in bronchioloalveolar cancer and adenocarcinoma [3]. Peripheral lung cancer mostly shows localized small nodules or patchy shadows in the early stage and is often misdiagnosed as inflammation or tuberculosis. As the tumor enlarges, it can form a higher density and rough edge nodular shadow with a diameter of 0.5∼1 cm. After the tumor diameter increases to 2∼3 cm, it may show a nodular shadow with increased density and clear boundary, accompanied by lobulation, umbilical fossa, or fine hair puncture [4].

As a solid space-occupying lesion in the lung, inflammatory pseudotumor of the lung is a chronic nonspecific inflammation in the lung caused by a combination of inflammatory cell aggregates and gradual fibrosis, which is similar to the clinical signs of lung cancer, tuberculosis, or other benign lung lesions [5–7]. Pulmonary inflammatory pseudotumor lacks specific clinical manifestations and imaging features and is easily misdiagnosed as lung cancer and tuberculosis and delays the diagnosis and treatment of patients [8]. With the improvement of people's health awareness and cancer prevention awareness, many patients diagnosed with small space-occupying lesions in the lungs choose surgical treatment, and a certain proportion of these space-occupying lesions are benign. Therefore, a diagnosis that can be accurate before treatment is most meaningful for patients.

CT technology has become the main means of early screening, diagnosis, and efficacy evaluation of lung cancer because of its simplicity, convenience, wide popularity, rapidity, and high efficiency. High-resolution CT can clearly show tumor lobulation, marginal spiculation, pleural indentation sign, and even calcium distribution type, bronchial inflation sign, and vacuole sign [9–11]. Although CT has been widely used in clinical practice, it is still easy to misdiagnose some benign lung lesions (pulmonary tuberculosis and pulmonary inflammatory pseudotumor) as peripheral lung cancer in clinical practice, resulting in unnecessary surgical treatment for patients and greater trauma to patients. Both peripheral lung cancer and pulmonary inflammatory pseudotumor are solid pulmonary masses, and the differential diagnosis on CT signs is difficult. At present, there have been many studies [12–16] that have compared the CT signs of the two diseases in an attempt to find the difference between the two. However, there were some differences in the conclusions of the investigators. Therefore, this study systematically evaluated the difference of CT signs of peripheral lung cancer and inflammatory pseudotumor by integrating the literature data between the investigators and performing the meta-analysis.

## 2. Materials and Methods

### 2.1. Literature Search

PubMed, Embase, Cochrane Library, CNKI, Wanfang, and CBM were searched to collect relevant studies on CT image comparison of peripheral lung cancer and inflammatory pseudotumor from database establishment to July 15, 2021. The searched languages were only Chinese and English. Search terms: “Lung Neoplasms”, “Pulmonary Neoplasms,” “Neoplasms, Lung,” “Lung Neoplasm,” “Neoplasm, Lung,” “Neoplasms, Pulmonary,” “Neoplasm, Pulmonary,” “Pulmonary Neoplasm,” “Lung Cancer,” “Cancer, Lung,” “Cancers, Lung,” “Lung Cancers,” “Pulmonary Cancer,” “Cancer, Pulmonary,” “Cancers, Pulmonary,” “Pulmonary Cancers,” “Cancer of the Lung,” “Cancer of Lung,” “Granuloma, Plasma Cell,” “Plasma Cell Granuloma,” “Granulomas, Plasma Cell,” “Plasma Cell Granulomas,” “Inflammatory Pseudotumor,” “Inflammatory Pseudotumors,” “Pseudotumors, Inflammatory,” “Pseudotumor, Inflammatory.” By PubMed database, the retrieval formula is:((((((((((((((((((“Lung Neoplasms”[Mesh]) OR (Pulmonary Neoplasms[Title/Abstract])) OR (Neoplasms, Lung[Title/Abstract])) OR (Lung Neoplasm[Title/Abstract])) OR (Neoplasm, Lung[Title/Abstract])) OR (Neoplasms, Pulmonary[Title/Abstract])) OR (Neoplasm, Pulmonary[Title/Abstract])) OR (Pulmonary Neoplasm[Title/Abstract])) OR (Lung Cancer[Title/Abstract])) OR (Cancer, Lung[Title/Abstract])) OR (Cancers, Lung[Title/Abstract])) OR (Lung Cancers[Title/Abstract])) OR (Pulmonary Cancer[Title/Abstract])) OR (Cancer, Pulmonary[Title/Abstract])) OR (Cancers, Pulmonary[Title/Abstract])) OR (Pulmonary Cancers[Title/Abstract])) OR (Cancer of the Lung[Title/Abstract])) OR (Cancer of Lung[Title/Abstract])) AND ((((((((“Granuloma, Plasma Cell”[Mesh]) OR (Plasma Cell Granuloma[Title/Abstract])) OR (Granulomas, Plasma Cell[Title/Abstract])) OR (Plasma Cell Granulomas[Title/Abstract])) OR (Inflammatory Pseudotumor[Title/Abstract])) OR (Inflammatory Pseudotumors[Title/Abstract])) OR (Pseudotumors, Inflammatory[Title/Abstract])) OR (Pseudotumor, Inflammatory[Title/Abstract])).

### 2.2. Inclusion and Exclusion Criteria

  Inclusion criteria: (1) the types of studies selected for this meta-analysis were retrospective studies; (2) the experimental group of the study was peripheral lung cancer and the control group was inflammatory lung pseudotumor; (3) the included studies needed to include at least one of the following indicators: lesion size, HU value of CT, HU value of enhanced CT, calcification, bronchial inflation sign, cavity, vacuole sign, pleural indentation sign, and burr sign; and (4) the reported data in the literature were complete.
  Exclusion criteria: (1) the results are not wholly statistically analyzed or relevant data are insufficient; (2) there is a repeated publication of literature; (3) the study subjects of literature are not patients with peripheral lung cancer and inflammatory pseudotumor of a lung; and (4) it is conference, meta-analysis, and review literature.

Two investigators first independently screened the retrieved literature according to the inclusion and exclusion criteria and then cross-checked them. The controversial literature was evaluated by the corresponding author and then unified through discussion. Two researchers extracted the relevant information of the included literature, mainly including the first author, publication year, publication country, sample size, lesion size, HU value of CT, HU value of enhanced CT, calcification, bronchial inflation sign, cavity, vacuole sign, pleural indentation sign, and burr sign.

The quality of the included articles was assessed by two investigators using the Newcastle–Ottawa (NOS) scale, a quality evaluation tool specifically for case-control studies and cohort studies. The evaluation included three aspects: selection (four items), comparability (one item), and outcome (three items). Among them, the maximum score of each item of choice and outcome was 1, the top score of comparable items was 2, and the total score of scale evaluation results was 9. Scores (0∼4) were classified as low-quality articles and (5∼9) as high-quality.

### 2.3. Statistical Methods

Meta-analysis of the data was performed using Stata 16.0 software, enumeration data were expressed as relative risk (RR), measurement data were expressed as the standardized difference (SMD), and interval estimation was described as 95% confidence interval (CI). Between-study heterogeneity was determined by the *χ*^2^ test combined with quantitative analysis of *I*^2^. If *P* > 0.1 and *I*^2^ < 50%, it was considered that between-study heterogeneity was acceptable, and a fixed-effect model was used for meta-analysis. If *P* < 0.1 and *I*^2^ > 50%, it was deemed that between-study heterogeneity was significant, and a random-effect model was used for analysis. The Egger test judged the publication bias of the included studies, and *P* > 0.05 indicated no significant publication bias.

## 3. Results

### 3.1. Literature Search and Screening Results

In this meta-analysis, 1662 relevant articles were obtained through preliminary retrieval, of which 869 remained after excluding repeated literature, 27 remained after excluding irrelevant study through the reading title, and eight remained after excluding literature, including abstract, animal study, and review through reading full text [12–16]. All were retrospective studies, including 4 English and 4 Chinese articles, involving 675 patients—literature screening procedure (Figure 1).

### 3.2. Basic Characteristics and Quality Assessment of Included Literature

Eight articles were included in this meta-analysis, and the basic characteristics of the studies are shown in Table 1. The quality of the included studies was evaluated. Four articles [12] had a NOS score of 5, 2 papers [14, 16] had a NOS score of 6, and 2 articles [13, 15] had a NOS score of 7. The quality assessment of all articles was ≧5 points, suggesting that the overall quality of the included articles was high.

## 4. Meta-Analysis Results

### 4.1. Lesion Size

Four pieces of literature reported the lesion size of inflammatory pseudotumor and peripheral lung cancer (Figure 2). The heterogeneity test was performed for the four included literature (*I*^2^ = 30.1%), indicating that the included studies had moderate heterogeneity. The fixed-effect model was used to combine the effect size. Meta-analysis showed that the lesion size of inflammatory pseudotumor was more significant than that of peripheral lung cancer, and the difference had statistical significance [SMD = 0.29, 95% CI (0.01, 0.58), *P* < 0.05].

### 4.2. HU Value of CT

Four pieces of literature reported the HU value of CT between inflammatory pseudotumor and peripheral lung cancer (Figure 3). The heterogeneity test was performed for the four included literature (*I*^2^ = 80.7%), indicating that the included studies had high heterogeneity. The random-effects model was used to combine the effect size. Meta-analysis results showed no significant difference in the HU value of CT between inflammatory pseudotumor and peripheral lung cancer [SMD = −0.09, 95% CI (−0.79, 0.60), *P* > 0.05].

### 4.3. HU Value of Enhanced CT

There were four pieces of literature in which the HU value of enhanced CT between inflammatory pseudotumor and peripheral lung cancer was reported (Figure 4). The heterogeneity of the four included literature was tested (*I*^2^ = 69.9%), indicating that the included studies had moderate heterogeneity. The random-effects model was used to combine the effect size. Meta-analysis results showed that the HU value of enhanced CT in inflammatory pseudotumor was higher than that in peripheral lung cancer, and the difference had statistical significance [SMD = 0.75, 95% CI (0.15, 1.34), *P* < 0.05].

### 4.4. Calcification

There were three literature pieces in which the incidence rate of calcification of inflammatory pseudotumor and peripheral lung cancer was reported (Figure 5). The heterogeneity test was performed for the included three pieces of literature (*I*^2^ = 0.0%), indicating no heterogeneity in the included studies. The fixed-effect model was used to combine the effect size. Meta-analysis showed that the incidence rate of calcification of inflammatory pseudotumor was significantly higher than that of peripheral lung cancer, and the difference had statistical significance [RR = 2.85, 95% CI (1.33, 6.11), *P* < 0.05].

### 4.5. Cavities

Four literature pieces reported the incidence rate of cavities of inflammatory pseudotumor and peripheral lung cancer (Figure 6). The heterogeneity test was performed for the four included literature pieces (*I*^2^ = 0.0%), indicating no heterogeneity in the included studies. The fixed-effect model was used to combine the effect size. Meta-analysis results showed no significant difference in the incidence rate of cavities between inflammatory pseudotumor and peripheral lung cancer [RR = 1.09, 95% CI (0.67, 1.78), *P* > 0.05].

### 4.6. Vacuole Sign

There were three literature pieces in which the incidence rate of the cavity of inflammatory pseudotumor and peripheral lung cancer was reported (Figure 7). The heterogeneity test was performed for the included three pieces of literature (*I*^2^ = 0.0%), indicating no heterogeneity in the included studies. The fixed-effect model was used to combine the effect size. Meta-analysis showed no significant difference in the incidence rate of vacuole sign between inflammatory pseudotumor and peripheral lung cancer [RR = 0.80, 95% CI (0.56, 1.15), *P* > 0.05].

### 4.7. Pleural Indentation Sign

Three pieces of literature reported the incidence rate of pleural indentation sign of inflammatory pseudotumor and peripheral lung cancer (Figure 8). The heterogeneity test was performed for the three included literature (*I*^2^ = 88.7%), indicating that the included studies had high heterogeneity. The random-effects model was used to combine the effect size. Meta-analysis results showed no significant difference in the incidence rate of the pleural indentation between inflammatory pseudotumor and peripheral lung cancer [RR = 0.42, 95% CI (0.15, 1.12), *P* > 0.05].

### 4.8. Burr Sign

Three pieces of literature reported the incidence rate of long hair puncture signs of inflammatory pseudotumor and peripheral lung cancer (Figure 9). The heterogeneity test was performed for the three included literature (*I*^2^ = 87.3%), indicating that the included studies had high heterogeneity. The random-effects model was used to combine the effect size. Meta-analysis results showed that the incidence rate of long hair puncture sign of inflammatory pseudotumor was lower than that of peripheral lung cancer, and the difference had statistical significance [RR = 0.49, 95% CI (0.24, 0.97), *P* < 0.05].

### 4.9. Bronchial Inflation Sign

There were three literature pieces in which the incidence rate of bronchial inflation sign of inflammatory pseudotumor and peripheral lung cancer was reported (Figure 10). The heterogeneity of the included three pieces of literature was tested (*I*^2^ = 41.9%), indicating that the included studies had moderate heterogeneity. The fixed-effect model was used to combine the effect size. Meta-analysis showed no significant difference in the incidence rate of bronchial inflation sign between inflammatory pseudotumor and peripheral lung cancer [RR = 0.94, 95% CI (0.69, 1.27), *P* > 0.05].

### 4.10. Sensitivity Analyses

Sensitivity analysis was required because of the significant heterogeneity in the four outcomes of HU value of CT, HU value of enhanced CT, the incidence of pleural indentation sign, and burr sign. No primary source of increased heterogeneity was found by the elimination method one by one. The results of the above four outcome measures were still relatively stable after excluding any study, indicating that the results of this meta-analysis were steady and reliable.

### 4.11. Publication Bias

Since a total of 8 literature pieces were included in this meta-analysis, the publication bias could not be effectively evaluated through a funnel plot. Egger's test was used to evaluate the lesion size, HU value of CT, HU value of enhanced CT scan surface, calcification, bronchial inflation sign, cavity, vacuole sign, pleural indentation sign, and burr sign, suggesting no significant publication bias in the above outcome indicators.

## 5. Discussion

This meta-analysis found that there were differences in some CT signs between peripheral lung cancer and inflammatory pseudotumors, inflammatory pseudotumors had larger lesions than peripheral lung cancer, patients with inflammatory pseudotumors had higher HU values and calcification incidences on contrast-enhanced CT than patients with peripheral lung cancer, and patients with inflammatory pseudotumors had a lower incidence of burr sign than patients with peripheral lung cancer. Therefore, lesion size, HU value of enhanced CT, calcification incidence, and burr sign may be important indicators for differentiating peripheral lung cancer from inflammatory pseudotumor, which has reference value for guiding clinical differential diagnosis.

The lung cancer of interest in this study is one of the most common diseases of the respiratory system. In contrast, inflammatory pseudotumors of the lung are rare benign lesions in clinical practice. Pulmonary inflammatory pseudotumor is an intrapulmonary mass caused by granuloma, fibrous connective tissue hyperplasia, and organization caused by chronic inflammatory lesions in the lung. The occurrence sites are mostly peripheral subpleural in the lungs, relatively rare in the left lobe, and there is no significant difference in the occurrence gender [17]. The shape of the mass is square mainly, generally accompanied by inflammatory infiltration blurred shadows in the periphery of the lesion, and a few are round and lobulated, mostly involving the adjacent pleura, causing local pleural thickening or pleural indentation, and even producing pleural effusion [18]. Most of the tumors showed significant severe enhancement after CT enhancement because inflammatory pseudotumor is a chronic nonspecific lesion with significant vascular proliferation, abundant, local formation of granulation tissue, significant enhancement after enhancement, and CT value increased by 60 HU; and most of the lesions showed delayed enhancement changes after enhancement, with clinical manifestations of cough, sputum, and even blood-stained sputum in severe cases, mainly in the middle and lower lobes and peripheral parts of the lung [19–21]. Peripheral lung cancer is a common clinical pulmonary malignant tumor characterized by lobulation sign, burr sign, vascular convergence sign, pleural indentation sign, and so on. There are many enlarged lymph nodes in the mediastinum and hilum. In severe cases, there are signs of pulmonary and distant metastasis. Most peripheral lung cancers have no apparent symptoms or specific characters in the initial stage. Most of them are found by physical examination and imaging examination, with early manifestations of fever and mild chest pain, and late symptoms such as face cervical oedema, hoarseness, and shortness of breath, with a low cure rate and a high mortality rate [20]. The clinical manifestations of pulmonary inflammatory pseudotumor and peripheral lung cancer alone cannot effectively distinguish the two, and it is necessary to use diagnostic instruments.

In this study, the lesion size of inflammatory pseudotumor was more significant than that of peripheral lung cancer, and the difference was statistically significant. The conclusion may be because the peripheral lung cancers compared by the investigators are early. After all, the peripheral lung cancers that are difficult to differentiate clinically are also primarily small. This study found no significant difference in HU values between inflammatory pseudotumor and peripheral lung cancer CT. In contrast, HU values were higher in inflammatory pseudotumor-enhanced CT than in peripheral lung cancer. It has been reported that the average CT of pulmonary inflammatory pseudotumor is 33.5 HU ± 6.66 HU, and it is speculated that there may be different degrees of oedema in inflammatory pseudotumor resulting in relatively low CT values. There are few reports on the significance of CT values. The enhancement findings of pulmonary inflammatory pseudotumor have been reported [22]. Some researchers found that, for 65 cases of arcuate noncalcified pulmonary nodules, with the injection rate of 4 ml/s and 100 ml of nonionic contrast agent, the CT value of inflammatory nodules increased quickly after contrast agent injection, with two peaks, the first average peak was about 36 s, the second average peak was about 100 s, and the size of the two mountains was similar, which were higher than those of the lung cancer group. Therefore, the results may be helpful for the diagnosis of pulmonary inflammatory pseudotumor [23].

In this study, we also found another valuable CT sign that inflammatory pseudotumor has a significantly higher incidence of calcification than peripheral lung cancer. Studies have demonstrated that lung cancer and inflammatory pseudotumors are mainly caused by lung inflammation. It is evident that the high incidence of calcification in inflammatory pseudotumors is easily understood with the involvement of more inflammatory cells during their development. The Burr sign is caused by thickening of pulmonary interlobular septa, vascular proliferation, and perilesional fibrosis due to inflammation or connective tissue production, and the burr sign can be seen as short and thin in patients with lung cancer. In contrast, the burr sign is longer and thicker in patients with pulmonary inflammatory pseudotumor. This is related to the difference in the pathological basis between the two. The former is due to the outward infiltration of cancer cells. The presence of cancer cells in some cells indicates that there will be a large number of inflammatory cells, lymphocytes, and fibrous connective tissue; the latter is due to the increased interlobular septa of the lung caused by inflammatory connective tissue and the surrounding fibres caused by vascular proliferation [24]. This study showed that the incidence of long hair spur signs in inflammatory pseudotumor was lower than in peripheral lung cancer, and the difference had statistical significance. This sign is also of great importance to differentiating peripheral lung cancer from inflammatory pseudotumor.

The results of this study showed no difference in the incidence of the cavity, pleural indentation, vacuole sign, and bronchial inflation sign in CT examination between patients with peripheral lung cancer and inflammatory pseudotumor. However, there were significant differences in the lesion size, burr sign, and incidence of calcification, indicating that, in the CT examination of peripheral lung cancer and inflammatory pseudotumor, careful attention to its characters is conducive to the differentiation of peripheral lung cancer and inflammatory pseudotumor. Although the data of this study showed no difference in intralesional cavities of lung cancer, according to previous data, its internal unsmooth in the signs of cavities of lung cancer lesions is in stark contrast to the smooth inner wall of inflammatory pseudotumor cavities, which has some differential diagnostic significance [25].

Although differential CT signs of some inflammatory pseudotumors and peripheral lung cancer were found, this study was limited by the original literature and failed to analyze the “knife-like changes” and lobulation of the mass. Inflammatory pseudotumors of the lung may be of great clinical value in the diagnosis of pulmonary inflammatory pseudotumors because they are pulled by fibrosis at the edge of the lesion, or the lesion along the edge of a lobe or segment may lead to knife-like changes with a straight and knife-like shape at one level in the middle of the lesion [21, 26]. Both inflammatory pseudotumor and peripheral lung cancer show lobulation, but peripheral lung cancer has more convex lobulation and deeper lobulation, and pulmonary inflammatory pseudotumor has only 19.51% lobulation and shallow lobulation [27]. In the past, the literature has proposed that the lobulation of the two is classified according to the chord length and arc-string distance ratio, of which deep lobulation is of great significance for the differential diagnosis between the two.

## 6. Conclusion

Although inflammatory pseudotumor and peripheral lung cancer have many similar CT features, careful identification of the two by HU value, lesion size, burr sign, and incidence of calcification on enhanced CT may be helpful for the differential diagnosis of the two, thereby reducing the misdiagnosis of patients and avoiding unnecessary treatment. Particularly in the state of the global outbreak of newly coronary pneumonia, the medical resources of respiratory diseases are relatively tight, and accurate diagnosis of pulmonary diseases will be necessary.

## Figures and Tables

**Figure 1:** Flowchart of literature search and screening.

**Figure 2:** Forest plot of the lesion size comparison between inflammatory pseudotumor and peripheral lung cancer patients.

**Figure 3:** Forest map of HU values of CT in patients with inflammatory pseudotumor and peripheral lung cancer.

**Figure 4:** Forest plot of HU values of enhanced CT in patients with inflammatory pseudotumor and peripheral lung cancer.

**Figure 5:** Forest plot comparing the incidence of calcification in patients with inflammatory pseudotumor and peripheral lung cancer.

**Figure 6:** Forest plot of the incidence of cavities in patients with inflammatory pseudotumor versus peripheral lung cancer.

**Figure 7:** Forest plot of incidence of vacuolation sign in patients with inflammatory pseudotumor versus peripheral lung cancer.

**Figure 8:** Forest plot comparing the incidence of pleural indentation sign in patients with inflammatory pseudotumor and peripheral lung cancer.

**Figure 9:** Forest plot comparing the incidence of long hair spur sign in patients with inflammatory pseudotumor and peripheral lung cancer.

**Figure 10:** Forest plot of incidence of bronchial inflation sign in patients with inflammatory pseudotumor versus peripheral lung cancer.

**Table 1:** Basic characteristics and quality evaluation results of the included literature.

Study	Year	Country	Type of study	Age (s)		Gender (M/F)		Sample sizes		Disease type		Outcomes	NOS scores
				Experimental	Control	Experimental	Control	Experimental	Control	Experimental	Control		
Xin et al.	2007	China	Cohort study	52 (31–73)	52 (31–73)	24/13	NA	37	104	Inflammatory pseudotumor	Peripheral lung cancer	(1)(2)(4)(5)(6)(7)(8)(9)	5

Zhao and Zheng [12]	2021	China	Cohort study	55.26 ± 1.48	55.26 ± 1.48	NA	NA	74	58	Inflammatory pseudotumor	Peripheral lung cancer	(4)(5)(6)(7)(8)(9)	5

Zhang et al.	2016	China	Cohort study	45.8 ± 1.5	47.3 ± 1.6	36/23	47/33	59	80	Inflammatory pseudotumor	Peripheral lung cancer	(4)(5)	5

Jing et al.	2021	China	Cohort study	45.35 ± 7.81	46.86 ± 8.22	25/16	21/13	41	34	Inflammatory pseudotumor	Peripheral lung cancer	(1)(3)(4)(5)(6)(7)(8)(9)	5

Hou et al. [13]	2014	China	Cohort study	62 (41–83)	62 (41–83)	NA	NA	25	35	Inflammatory pseudotumor	Peripheral lung cancer	(1)(3)	7

Xie [14]	2011	China	Cohort study	19–55	34–77	4/6	22/14	10	36	Inflammatory pseudotumor	Peripheral lung cancer	(2)(3)	6

Wang and Shan [15]	2017	China	Cohort study	54.6 ± 14.3	60.7 ± 12.1	6/10	22/16	16	38	Inflammatory pseudotumor	Peripheral lung cancer	(1)(2)	7

Zhang et al. [16]	2002	China	Cohort study	47 (37–78)	58 (40–75)	4/3	11/10	7	21	Inflammatory pseudotumor	Peripheral lung cancer	(1)(2)(3)	6

## Data Availability

The simulation experiment data used to support the findings of this study are available from the corresponding author upon request.
